The article "Analysis of the Natural Conditions and Geographical Factors of the Formation of Hui-Style Prints" was retracted in 2023. Reasons: unreliable results or conclusions; concerns about the data; concerns about the peer review; concerns about the citations.

# Analysis of the Natural Conditions and Geographical Factors of the Formation of Hui-Style Prints

**DOI:** 10.1155/2022/4627215

**Published:** 2022-07-14

**Authors:** Shangke Li

**Affiliations:** School of Art and Design, North China University of Water Resources and Electric Power, Zhengzhou 450000, China

## Abstract

In order to analyze the natural conditions and geographical factors of the formation of Hui-style prints, big data analysis technology is brought in, through which more audiences can understand the true meaning of Hui-style printmaking, the internal system of Hui-style printmaking during its operation can be improved, and artists can complete the analysis of natural conditions and geographical factors for the formation of Hui-style prints by means of empirical analysis. In this way, during the implementation of artistic acts, the benefits of the city and even the society can be increased, and the social and economic benefits can be improved accordingly and involved in information management systems directionally, and the natural conditions and geographical factors related to the formation of Hui-style prints can be deeply analyzed, so as to ensure that the formation of Hui-style prints has a social and economic promotion.

## 1. Introduction

With the continuous improvement of China's economic benefits, the government and relevant departments have gradually increased their attention to art and culture [1]. In this context, in order to control the pace of urbanization, we should pay more attention to the formation of Hui-style prints, pay attention to natural conditions, and analyze them in combination with geographical factors. Through the setting of categories during the formation of Hui-style prints, the statistical work of data in all aspects is improved (as shown in Figure 1).

From this point, we can confirm that the formation of Chinese Huizhou printmaking can be smoothly promoted, so that art creators can master the basic characteristics of the region. At the same time, through the understanding of Huizhou region, the natural landscape of Huizhou region can be reflected in printmaking. For example, the four wonders of Huangshan that are the sea of clouds, hot springs, grotesque rocks, and pines. Artists can analyze the actual landscape of the Huizhou area and master the area with beautiful scenery so as to ensure that it can be viewed in the mountainous area of southern Anhui [2]. In this way, both the magical landscape and Qiyun rock and gully can be seen by artists to ensure that their Hui-style prints can be called a great story. On this basis, the formation of Hui-style prints is affected by economic and social benefits, resulting in increased interference factors in the formation of Hui-style prints, which is also harmful to the creation of artists. Therefore, all departments gradually realized the seriousness of this problem and gradually increased their attention to the formation of Hui-style prints [3].

At this point, the natural conditions and geographical factors for the formation of Hui-style prints are taken as the background, and the application in the formation of Hui-style prints is also planned by category and time so as to ensure that the formation of Hui-style prints can meet the aesthetic requirements of artists and promote social and economic development (as shown in Figure 2) [4].

In this way, it can be calculated that geographical factors play a role in the formation of Hui-style prints, increase the favorable factors for artists in the design of works, and ensure that the comprehensive aesthetic consciousness of local people and even the citizens of each region can be improved accordingly, which can improve the quality of people's lives and enrich the content of people's daily life [5].

## 2. Research Significance

In the analysis of the natural conditions and geographical factors of the formation of Hui-style prints, we can focus on the analysis of social development and the ability to achieve economic benefits in the Huizhou area. First of all, we can use big data analysis to grasp the basic trend of local economic development and social development and give corresponding auxiliary factors in the formation process of Hui-style prints through the Huizhou area. As a result, the author thinks that the analysis can be carried out from an economic perspective to ensure the reasonable construction of the communication system during formation of Hui-style prints to ensure that the basic performance of the formation of Hui-style prints can be highlighted in the computer system, to complete the analysis of natural conditions and social factors, and to ensure that the formation of Hui-style prints can promote the local economic benefits [6].

Secondly, it can elaborate on the formation of Hui-style printmaking, paving the way for artists' cultural creation and ensuring that the formation of Hui-style printmaking can meet artists' pursuit of beauty so as to ensure that the formation of Hui-style printmaking can play a corresponding boosting role. At the same time, in terms of environmental conditions, artists can learn the connotation of Hui-style printmaking during its formation, pay attention to its potential elements in the development process, and ensure that the formation of Hui-style printmaking is more meaningful through continuous innovation and development. If we cause the formation of Hui-style printmaking and the development of Huizhou to connect closely, a complete guarantee mechanism can be built, and corresponding assistance to the cultural development of Huizhou can be provided [7]. Therefore, the author thinks that we can combine the geographical factors and natural conditions of the Huizhou area to analyze and understand the historical process of this area and make the tourists who pass through the Huizhou area fall in love with the Huizhou culture so as to ensure that they can fall in love with the quiet landscape and have the idea of living in this area for a long time.

In this way, the favorable factors in the formation of Hui-style prints can be increased. With the long-term efforts of artists from various departments, the complete artistic expression forms will be highlighted, and Hui-style prints will be endowed with a certain sense of history and the times so that the artistic style of Hui-style prints is more obvious not only in techniques to exist but also in style to be reflected, whose purpose is to improve the system structure of Hui-style printmaking during its formation, to promote the further development of national culture, then to make Hui-style printmaking become the main line of Chinese printmaking art, and finally to make it reflect the basic connotation of poetic painting during its formation [8].

## 3. Literature Review

Depending on the development process of the times, contemporary people's demand for beauty is gradually increasing, resulting in the formation of Huizhou printmaking as an indispensable cultural supplement in the daily life of Huizhou [9]. At the same time, nowadays, the number of different kinds of artworks is increasing year by year. If people ignore the consideration of national culture in the Huizhou area, it will restrict the development of art and culture in the Huizhou area, lead to the formation of Hui-style printmaking, and increase the adverse factors for the development of the environment in the Huizhou area. Therefore, in order to ensure that Hui-style printmaking is closer to the process of the times, the formation mode of original Hui-style printmaking can be innovated so that it is not limited to geographical factors and natural conditions but can increase the interference of human factors. Big data analysis, intelligent technology, cloud computing, and other related technologies should be used to add auxiliary factors during the formation of Hui-style prints so that local people can correctly understand the formation significance of Hui-style prints. Under this background, the connotation of national culture in Huizhou can also be highlighted through the formation of Hui-style prints [10].

Meanwhile, the principle of superposition can be used to analyze and interpret the formation mode of Hui-style prints. Instead of using single small crack stress, intensity factor *K* and crack opening displacement can be applied to realize the analysis of natural conditions during the formation of Hui-style prints and to ensure that there will not be too many position variables during the formation of Hui-style prints, causing the artists to combine their own development trends for analysis to achieve the detection of the whole Huizhou. Finally, the analysis of the natural conditions and geographical factors for the formation of Hui-style prints is then completed, which can reflect the basic connotation of national culture [11].

## 4. Methods

### 4.1. Research Schemes to Solve the Problems

#### 4.1.1. Identify the Natural Conditions for the Formation of Hui-Style Prints

In terms of the formation of Hui-style printmaking, because the Huizhou area is located in the mountainous area of southern Anhui, it has the characteristics of relatively weak real estate, more local mountainous areas, and fewer fields [12]. If only the natural environment is analyzed, the smooth formation of Hui-style prints during this period will not be guaranteed, and the increasing influence of the natural environment on Hui-style prints leads to the phenomenon that most painters struggle with nature and strive for survival advantages. Therefore, the application of big data analysis technology in this stage can be increased to let more artists know the main forms of Hui-style printmaking by means of picture expression so as to ensure that natural conditions can give full play to their role in the formation of Hui-style printmaking (as shown in Figure 3) [13].

In the long run, the formation of Hui-style prints has corresponding characteristics, but most of them are based on the geographical characteristics of the Huizhou region [14]. Therefore, in order to complete the analysis of the natural conditions during the formation of Hui-style prints, the natural influencing factors in the area can be applied to the work of printers, painters, engravers, and bookstore employees, which enables artistic creation activities to be carried out smoothly, so as to ensure that artists in different regions can increase the favorable factors in the formation process of Hui-style printmaking according to their own development, so as to ensure that each artist can go his own way and get a better competitive space in the natural environment (as shown in Figure 4).

As shown above, the addition of different natural environmental factors (*N*) can ensure that artists can innovate their professional abilities during the process of Hui-style printmaking and ensure that each artist can have the corresponding research spirit so that they can use distinctive artistic creation methods to complete various tasks [15]. At the same time, the vertical formula can be substituted by using data analysis:

(1) $$\begin{array}{c} N=\text{S}\cdot \text{t}\sum_{j}^{n}\beta j. \end{array}$$

Here, *s* is a variable constant, *t* is the time, *β* is the intercept of relevant data in the computer system, *j* is the dynamic change value, and *n* is the uncertainty factor in the computer system. In this way, the traditional values of *β* can be determined to ensure that the parameters of all aspects can be proportional to the state. Meanwhile, the dynamic planning influence brought by natural environmental factors during the formation of Hui-style prints can be planned as described in the following formula:

(2) $$\begin{array}{c} Y1=\beta 0+x\beta +\xi *J. \end{array}$$

In this way, regression parameters in Hui-style prints will not be affected by other factors; according to the influence of natural conditions, a linear regression model is created, the core points of Hui-style prints during their formation are confirmed, and it can be ensured that the research work of various data can be carried out normally, the induction and integration of internal variable factors and immutable factors can be promoted, and the method of regression estimation of parameters can be used:

(3) $$\begin{array}{c} \beta =\left(n^{x}n^{y}\right), \end{array}$$

where *n* is the minimum value in binary classification and *x* and *y* are the normal variables of regression parameters. At this point, we can ensure that Hui-style prints can be formed smoothly in the natural environment by means of data analysis in all aspects so as to increase the favorable factors for artistic creators during the implementation of various works [16]. In addition, the data change data in Figure 5 can be used for analysis to ensure that

(4) $$\begin{array}{c} A=\frac{a}{\left(2R\right)}. \end{array}$$

Here, *a* mainly represents the stress intensity of Hui-style prints in the natural environment, while *R* represents the three-point bending sample in the drawing area of Hui-style prints in different degrees. As shown in Figures 6or 7, the eccentricity distance of different loads during the formation of Hui-style prints can be measured to ensure the smooth development of each sample [17, 18].

At the same time, the favorable factors during the formation of Hui-style prints can be increased to have the disks containing single/bilateral cracks connected by means of docking when the artists are drawing their different works to ensure that the radial concentration force *P* inside can be applied to each area, to complete the detection of infinite steel stress, and to control the strength factors in the formation stage of Hui-style printmaking to promote the operation of artists to be more standardized and analyze the deficiencies in the formation stage of Hui-style printmaking so that the double cracks and single cracks can be more intuitively shown (as shown in Figure 8) [19, 20].

#### 4.1.2. Confirm Social Factors in Hui-Style Prints

In order to determine the natural conditions and geographical factors that existed during the formation of Hui-style prints, it is necessary to increase the application of big data algorithm through experimental analysis, master the data information existing during the formation of Hui-style prints by using the input stage, and then record all aspects of information in the reader, to complete the editing of the file information, whose purpose is to enable every piece of data to be edited and sorted out by the computer system to complete the analysis of data and control the key values in the computer [21, 22]. In this way, all aspects of data can be guaranteed to be included in the mapper, facilitating the formation of vigorous vitality in Hui-style prints. Thus, geographical factors and natural conditions can be analyzed through computer software (as shown in Figure 9).

At that time, the internal functions of Hui-style printmaking can be defined through the computer system. Through a series of key values, the data in the system process will be processed, and zero or more key values will be generated to make sure that the middle key can generate the corresponding prime value based on geographical conditions and natural environmental factors, enable the combiner to combine all aspects of information in the system, ensure that it can show all aspects of data in the same area, and complete the mapping of small range values through the mapper in the form of code (as shown in Figure 10) [23, 24].

At the same time, to ensure that there will not be too many influencing factors in the formation of Hui-style prints, the unknown variable N can be used for the calculation, the strength factor is set to *k*, and then *U* is the crack tension displacement, which makes the artists think that the unknown variable in the formation process of Hui-style print has not been measured. Using the form of (*N* + 2) to perform the operations and using the equations of (*N* + 2) to embody the basic conditions of a crack in the practical work of link effect, the equation can be set up as follows:

(5) $$\begin{array}{c} \left\{U\left(1,x\right)=0;\right.\;x=\left(x1+xn+1\right);\;n=1,2,3\ldots ,N. \end{array}$$

Secondly, it can be analyzed in combination with the formation process of Hui-style printmaking to confirm that the setting mode of the equation is relatively complete and increase the application of continuous distributed stress in the computer software system. Through big data analysis, each stress that can be evenly distributed in the discrete form should be ensured, loopholes in the actual operation should be reduced, and then the following equation is ensured:

(6) $$\begin{array}{c} k=0. \end{array}$$

Thirdly, according to the displacement of elastic ligament in the computer system, it can be integrated to ensure that all data at *N* point can run in the direction of 0. The integration of love *N* is appropriately increased to reduce the frequency of discrete problems and promote the connectivity in the plastic region. At this point, the equation can be confirmed as follows:

(7) $$\begin{array}{c} \left\{\begin{array}{c} k=0,\\ U\left(i,0\right)=0, \end{array}\right. \end{array}$$

where *U* mainly represents the critical region of unknown quantities and the value represented by *i* in the way of load compliance is confirmed to avoid the appearance of outer cracks in the formation of Hui-style prints so that artists can analyze the geographical characteristics of Huizhou and increase the favorable factors in the formation of Hui-style prints. The external load and opening displacement during the formation of Hui-style prints show a coordinated state, and then the actual curve is distributed to ensure the formation of Hui-style prints under the action of natural conditions and geographical factors.

### 4.2. Test Method of Validation Scheme

#### 4.2.1. Weighting Function Method in Natural Conditions

Based on the analysis of the national cultural characteristics of the Huizhou area, the residual strength in the process of the formation of Hui-style printmaking is determined by the weight function method in natural conditions so as to ensure the normal operation of all analysis operations and avoid mistakes when artists are drawing and ensure that the method of improving the yield band is used. The formation model of Hui-style printmaking is established in the natural environment, and folk customs and related cultural contents are integrated to ensure that the formation of Hui-style printmaking can be applied under the external load to realize the improvement of Hui-style printmaking in the initial stage, to control the pressure in the computer system, to ensure the reasonable application of all data, and then to express through the form of equations:

(8) $$\begin{array}{c} \left\{\begin{array}{c} \varsigma \left(a0,a0\right)=\varsigma 0;\\ \varsigma \left(a,a=d\right)=2\;d\;\tan\left(\frac{a0}{2}\right)+\varsigma 1\left(a-d,a-d\right). \end{array}\right. \end{array}$$

In the formula, *a* − *d* exists as the actual tension of Hui-style prints, in which *a* and *b* can be planned as the basic variable, and then *ς* is the random quality; in the process of artistic creation, artists only need to measure the tension angle to master the influence of natural conditions and geographical factors on the formation of Hui-style prints. Under this background, the smooth development of crack propagation can be guaranteed to realize the integration of various data within the computer system, control the defects existing in the finite width plate and collinear crack, and ensure that the setting of the model is more reasonable and compliant [25].

#### 4.2.2. Backward Weight Function Method in Geographical Factors

In the formation period of Hui-style prints, it is necessary to increase the consideration of various aspects, and the inverse weight function method in geographical factors can be used to determine so as to ensure the smooth development of computational convergence, to increase the application of program algorithms during this period so that the residual strength of all aspects can be consistent with the process of Hui-style print formation, and then the solution program and finite element method are used to ensure that the inverse weight function method can be applied to the calculation of different number sets. In this way, the stress borne by Hui-style prints during construction can be analyzed by using the equation:

(9) $$\begin{array}{c} f\left(x\right)=\varsigma +\sum_{m=1}^{\infty }\left(m\;\cos\frac{a\pi x}{L}+\varsigma \;\sin\frac{a\pi x}{L}\right). \end{array}$$

In formula (9), *m* exists as the exact value of direction solution during the formation of Hui-style prints, while *L* is the concentrated stress. In this way, artists can detect all the data during the formation of Hui-style prints by using the reverse weight function method and store all the data information in the system through collection, retrieval, and processing to ensure that the elastic mechanics value under concentrated stress is more accurate and to ensure the integrity of the data. At the same time, it can be analyzed through data shown in Table 1.

It can be seen from Table 1 that, after the application of the inverse weight function method, data in all aspects tend to be stable. However, without the addition of the inverse weight function method in Table 2, the change trend is not stable enough.

Therefore, in order to control the formation state of Hui-style printmaking, the application of inverse weight function method can be increased, the dynamic programming problem can be rationally planned so that the accuracy of data in all aspects can be guaranteed, and the favorable factors in the formation process of Hui-style printmaking can be increased. Under this background, the equation can be listed in the way of likelihood function:

(10) $$\begin{array}{c} \text{PLR}=-\sum_{i=1}^{N}\left\{yi\;\ln\;\pi 1+\left(1-yi\right)\ln\left(1-\pi \right)\right.. \end{array}$$

According to formula (10), through the detection of the formation factor (*y*) of Hui-style printmaking, the state of variable factor *n* can be confirmed under specific circumstances, and the operating state of the changing parameters of system *i* can be mastered to avoid errors during actual operation. In this way, PLR status can be changed according to actual variables through the estimation so as to ensure that Huizhou engraving can be used as the basic factor for the formation of Hui-style printmaking so that people in this area can draw specific folk key points according to their own strengths. For example, in the early years, there were 4175 books written by scholars on the history of Huizhou, most of which were about the local cultural characteristics, folk customs, and cultural characteristics. However, the data are few, and the actual number of books written remains to be further studied. Therefore, in order to ensure that the natural conditions and geographical factors for the formation of Hui-style prints can play a certain auxiliary role, we can analyze the cultural relics, ancient collections, books, and related historical products in the Huizhou area to realize the rectification of the work content of book carving industry, to promote the formation of Hui-style printmaking more meaningful, and to ensure that these factors can give corresponding auxiliary support to the staff of artistic and cultural works; what is more, we should adhere to the basic concept of seeking truth and being pragmatic and control the cost consumption in the production of cultural and artistic products in all aspects to avoid too many problems during the formation of Hui-style prints. In this way, people are fully aware of the importance of the formation of Hui-style prints, and people in Huizhou are also aware of the profitability of fashionable industries, which lead to the rise of new cultural industries.

In this background, namely, if the smooth formation of Hui-style prints can be guaranteed, the development of shops in Huizhou will be increased to ensure that the working ability of each department is improved accordingly to ensure that there is evidence for the formation of Hui-style prints. The supplementary factors in operation and management should be added to enable the cultural color of Huizhou to be displayed in the network environment and social environment in order to promote the economic development of the Huizhou area and to let local people become richer so that they can rely on relatively strong financial resources and the development of Huizhou printmaking related industries, promote the rise of local book carving industry in Huizhou area in today's society, and promote the further development of Huizhou printmaking.

## 5. Results

The natural conditions and geographical factors of the formation of Hui-style prints can be analyzed according to the current development mode of economic benefits within the society; the way of evaluation can be used to ensure the reasonable construction of the development system of Hui-style prints; the means of empirical analysis can be used to ensure that artists can stand in multiple perspectives to think, strengthen the analysis in multiple aspects to ensure that the current situation of the development of Huizhou commerce is reasonably analyzed and Huizhou newspapers can be used as a predecessor of the formation of Hui-style prints, and then highlight the advantages of the Huizhou area through a variety of ways to analyze the formation of Hui-style prints.

As far as the Huizhou area is concerned, its local folk customs have unique characteristics in the expression process of literary and artistic works, perhaps with some local flavor, highlighting the characteristics of strong local and mellow folk flavor. Therefore, in the process of expressing folk customs and habits in the Huizhou area, more attention should be paid to artistic works, and the form of feedback should be used to highlight the basic forms of expression during the formation of Hui-style prints. In this way, Huizhou folk customs can be guaranteed to exist as an objective subject. At this time, in order to ensure the smooth development of cultural creation, artists need to increase the application of production and life elements. The natural conditions for the formation of Hui-style prints can meet the aesthetic needs of artists for cultural works, reduce the differences of ethics in cultural creation, and highlight local conditions and practices through the repetitive and regular basic expression forms and the development of cultural activities with periodic significance. Under this background, the expression of folk custom can be realized so that it can take on the form of branding and enrich the artistic factors during the formation of Hui-style prints, and then it gradually becomes a unique art and culture in the lives of working people, causing people in daily life to reflect the aesthetic interest and to show the fine connotation of a nation.

As there are certain differences in people's life links, there may be more differences in a nation or a region, but as long as there are people living here, there will be folk arts and folk customs. Therefore, the formation of Huizhou folk customs can also be called the crystallization produced in the long-term development process of people in the Huizhou area. If we analyze it from the perspective of history, the budget for the formation of Hui-style prints will be realized. At first, the artistic color of the life of the Huizhou people can be added, and the Hui-style printmaking formed by natural conditions can be ensured by analyzing the mountain customs such as “break the body.” Secondly, some people in the Huizhou area moved from the central plains and northern areas. Under the influence of history, the local basic folk customs will change qualitatively, and Huizhou customs with folk characteristics will be formed through migration or emigration. In this way, both the formation of Hui-style prints and the changes in local folk customs are closely related to natural conditions. At this time, this change exists as a new custom, which can keep the characteristics of the ancient Yue people forever, facilitating the current people in Huizhou to carry forward the local folk customs so that artists can abandon bad customs and habits, and the new Huizhou customs to create can be used to complete the calculation of the formation of Hui-style prints; therefore, it is convenient for people to consider from different dimensions and realize the discussion of various aspects of data results during the formation of Hui-style prints.

The formation process of Hui-style printmaking can be regarded as the evolution process of folk customs and national culture in the Huizhou area, which evolves from the aspects of language and customs, resulting in corresponding changes in culture, art, folk art, and handicrafts in the Huizhou area. Therefore, the formation of Hui-style prints can exist as a constantly changing process, and we can analyze it from the grassroots level to understand the basic expression of the ethnic art in the Huizhou area and take passion and joy as the creation theme of Hui-style prints through subject innovation, art rectification, and innovation. For example, through folk art themes such as Fu Lu Shou Samsung, the characters arrangement and story content arrangement are used to enrich the content of Hui-style printmaking so that posters and dramas are included in the creation category of Hui-style printmaking, such as The Empty City Plan. In this way, through the characteristics of the times, the spiritual outlook of historical figures can be displayed, the geographical factors of the Huizhou area can be highlighted, and the geographical factors can be included in the formation process of Hui-style prints so that the style can be shifted from the previous period of the relatively convergent art theme to the direction of bold and unrestrained change. On this basis, on the one hand, the inheritance of traditional culture can be realized; on the other hand, the formation process of Hui-style prints can reflect the folk customs of the Huizhou area.

Finally, it can be analyzed according to the formation mode of Huizhou folk prints to master the historical retained treasures in the Huizhou area and to ensure that the development of folk activities will not be restricted by external factors so that the formation of Hui-style prints will be more meaningful, the masses will be stabilized, and the enthusiasm of folk artists to create Hui-style prints will be mobilized.

## 6. Conclusion

Through the formation of Hui-style prints, the application of natural conditions and geographical factors can be added to have all aspects of folk customs data in the Huizhou area sorted into the formula calculation link so as to ensure the formation of Hui-style prints more accurately. Through the comprehensive evaluation method, all aspects of the data in the formation of Hui-style prints are edited, sorted, and stored in the computer software system to complete the analysis of the cost and creation data during the formation of Hui-style prints. By substituting the geographical factors in the formation of the Huizhou edition with the method of inverse weight function, the basic representation of folk customs in the Huizhou area can be highlighted, and the aesthetic consciousness of people in this area can be improved. To sum up, in order to create excellent Hui-style prints, it is necessary to attach importance to natural conditions, add folk customs, folk customs, and even national elements in the Huizhou area, and pay more attention to local geographical factors so as to ensure that the formation of Hui-style prints has unique art culture and promote the better development of Huizhou area.

## Figures and Tables

**Figure 1:** Hui-style print formation comparison chart of categories and time.

**Figure 2:** Added natural condition categories and time plan maps.

**Figure 3:** Hui-style print formation diagram of the link of big data analysis and determination.

**Figure 4:** Influence of natural conditions on the formation of Hui-style prints.

**Figure 5:** Hui-style print changes in binary classification in natural environment.

**Figure 6:** Stress intensity curve of Hui-style printmaking in natural environment.

**Figure 7:** Stress variation of Hui-style print in natural environment.

**Figure 8:** Variation of intensity factors in Hui-style prints.

**Figure 9:** Use computer to adjust the flowchart of Hui-style print.

**Figure 10:** Hui-style print in the data group identification layout.

**Table 1:** Hui-style prints in the inverse weight function method to add change data.

Serial number	Minimum value	Maximum value
1	+9.26%	+15.00%
2	+8.00%	+13.56%
3	+3.02%	+4.00%

**Table 2:** Natural variation data in Hui-style prints.

Serial number	Minimum value	Maximum value
1	+13.25%	+16.00%
2	+12.59%	+18.56%
3	+9.00%	+14.00%

## Data Availability

The labeled dataset used to support the findings of this study is available from the corresponding author upon request.
